The article "Classification and Drug Resistance Analysis of Pathogenic Bacteria in Patients with Bacterial Pneumonia in Emergency Intensive Care Unit" was published in 2022. Journal: Contrast Media Mol Imaging.

# Classification and Drug Resistance Analysis of Pathogenic Bacteria in Patients with Bacterial Pneumonia in Emergency Intensive Care Unit

**DOI:** 10.1155/2022/6980091

**Published:** 2022-09-30

**Authors:** Kai Yin, Ling Liu, Guofeng Fan

**Affiliations:** ^1^Department of Emergency, Nanjing Drum Tower Hospital, The Affiliated Hospital of Nanjing University Medical School, Nanjing 210008, China; ^2^Department of Pneumology, Nanjing Drum Tower Hospital, The Affiliated Hospital of Nanjing University Medical School, Nanjing 210008, China

## Abstract

**Objective:**

This study aimed to compare the identification efficiency of metagenome next generation sequencing (mNGS) and traditional methods in detecting pathogens in patients with severe bacterial pneumonia (BP) and further analyze the drug resistance of common pathogens.

**Methods:**

A total of 180 patients with severe BP who were admitted to our hospital from June 2017 to July 2020 were selected as the research objects. Alveolar lavage fluid from the patients were collected, and pathogens were detected by the mNGS technology and traditional etiological detection technology. Common pathogens detected by mNGS were tested for the drug sensitivity test. The difference between mNGS and traditional detection method in the identification of pathogenic bacteria in severe BP patients was compared, and the distribution characteristics and drug resistance of pathogenic bacteria were analyzed.

**Results:**

The positive rate of mNGS detection was 92.22%, which was significantly higher than that of the traditional culture method (58.33%, *P* < 0.05). 347 strains of pathogenic bacteria were detected by mNGS, including 256 strains of Gram-negative bacteria (G^−^), 89 strains of Gram-positive bacteria (G^+^), and 2 strains of fungi. Among G^−^ bacteria, *Acinetobacter baumannii* had higher resistance to piperacillin/tazobactam, ceftazidime, imipenem, levofloxacin, amikacin, ciprofloxacin, gentamicin, and the lowest resistance to tigecycline. The resistance of *Klebsiella pneumoniae* to piperacillin/tazobactam and ceftazidime was higher. *Pseudomonas aeruginosa* had low resistance to all the drugs. Escherichia coli had high drug resistance to most drugs, and the drug resistant rates to cefoperazone/sulbactam, piperacillin/tazobactam, ceftazidime, imipenem, and gentamicin were all more than 50.00%. G^+^ bacteria had high resistance to penicillin, azithromycin, amoxicillin and levofloxacin, and amoxicillin and levofloxacin had high resistance, up to 100.00%.

**Conclusion:**

mNGS has high sensitivity for the identification of pathogenic bacteria in patients with BP. G^−^ bacteria were the main pathogens of BP, but both G^−^ and G^+^ bacteria had high resistance to a variety of antibacterial drugs.

## 1. Introduction

Bacterial infection causes bacterial pneumonia (BP) most often, accounting for about 80%. The common symptoms are chest pain and cough. If drug intervention is not given in time, BP will progress to severe BP, and the patients will show serious adverse clinical symptoms such as high fever, dyspnea, and pulmonary respiratory failure, threatening the life safety of patients [1, 2]. Although BP has a good prognosis, with the change of pathogen spectrum, the clinical symptoms gradually tend to be “atypical,” which increases the difficulty of treatment and is easy to develop into refractory pneumonia. Severe BP has a high fatality rate in children, the elderly, and immunosuppressed patients, which should be paid attention to [3]. At present, antibiotics are the main means of clinical treatment of severe BP, but different pathogens have different drug resistance to antibiotics [4]. Some studies have found that the primary elected antibacterial agents for treating severe BP patients are associated with the prognosis of the disease to a certain extent, but most patients receiving primary treatment empirically, resulting in unreasonable use of antibacterial drugs, the gradual increase of drug-resistant bacteria and the variety of bacteria species, which brings certain difficulties for clinical treatment of the disease [5, 6]. The radical treatment of severe BP needs to start from the control of the distribution of pathogenic bacteria in patients because the number and distribution of pathogenic bacteria directly affect the severity of pneumonia in patients. With the progress of medical technology and the accumulation of experience of doctors, how to timely prevent, diagnose, and treat patients with severe BP has become a hotspot of clinical research at present [7, 8]. With the development of modern medicine, the variety of antibiotic drugs is increasing, and the number of drug-resistant bacteria is also increasing, which brings great challenges to clinical drug intervention. Therefore, how to detect pathogens quickly and accurately, and how to accurately grasp the epidemiological distribution and drug resistance of pathogens are the key to effective infection control. However, there is still a lack of clinical studies on the precise distribution and drug resistance of pathogenic bacteria in severe BP patients. Hence, 180 patients with severe BP admitted to our hospital from June 2017 to July 2020 were selected as the subjects of this study. Alveolar irrigation fluid of patients was obtained for microbial culture and NGS detection, aiming to analyze the pathogen status and drug resistance of patients with this disease and provide reference for clinical treatment of patients with severe BP [9].

## 2. Materials and Methods

### 2.1. Subjects

A total of 180 patients with severe BP diagnosed in our hospital from June 2017 to July 2020 were selected. The confirmed patients met the relevant standards in the Expert Consensus on Clinical Practice of Emergency Severe Pneumonia in China [10] and underwent laboratory and imaging examination, with no other infectious diseases, with good communication skills, and with ideal degree of coordination. Exclusion criteria for included patients are as follows: pregnant women: those with abnormal coagulation function; those with allergic constitution; those complicated with malignant tumor; those with renal insufficiency; those with impaired liver function; those with infectious diseases; and those with severe deficiency of immune system (e.g., HIV infection and posttransplant immunosuppression). Basic information is shown in Table 1.

### 2.2. Research Methods

#### 2.2.1. Alveolar Lavage

The next generation sequencing (mNGS) technique and traditional pathogen detection technique were used for pathogen detection. All patients underwent alveolar lavage after admission, and 2 portions of alveolar lavage fluid, 10–20 mL each, were taken at the same time. One was sent for traditional etiological examination (bacterial culture and fungal culture) and the other was tested for metagenomic NGS (mNGS).

#### 2.2.2. Biochemical Identification and Drug Sensitivity Test of Bacteria

Qualified specimens were collected on the blood plate, chocolate medium, and McConkey for culture at 35°C overnight. The isolated strains were identified by Vitek 2 compact system. The results were judged by CLSI standard execution.

#### 2.2.3. Detection Method mNGS Detection

The alveolar lavage fluid of the patient was sequenced by the Beijing Genomics Institute (BGI), and the samples were separated, extracted, and purified after examination. The library was prepared by DNA fragmentation, terminal repair, sequencing connector connection, and PCR amplification, and then it was sequenced by the machine. Then, artificial intelligence analysis was carried out to accurately identify pathogenic microorganisms. Authoritative clinical microbiology experts and clinical experts set the weight matrix of the database according to long-term clinical experience and global clinical testing standards and conducted automatic and rapid analysis and interpretation based on the weighted election-based horizontal labeling method.

Traditional detection: the alveolar lavage fluid samples of the patients were sent to the clinical laboratory of our hospital for smear and culture testing.

### 2.3. Observation Targets

(1) The distribution of pathogenic bacteria of the samples detected by mNGS and traditional detection method; (2) drug resistance of main G^−^ bacteria; and (3) drug resistance of main G^+^ bacteria.

The criteria for positive results by mNGS are as follows: (1) microorganisms were identified by both traditional detection method and mNGS; (2) imaging manifestations of pulmonary lesions; (3) if the microbial readings obtained by the high-throughput assay were at least two times higher than those of other microorganisms, the identified microorganisms were classified as confirmed pathogens. Microorganisms identified by mNGS alone and in line with (1) and (2) were considered as new potential pathogenic microorganisms.

### 2.4. Statistical Method

SPSS 23.0 statistical software was used to analyze the data. The counting data were expressed as percentage (%). The difference was compared by *χ*^2^ test, and the paired chi-square test (McNemar's test) compared the difference of the paired data.

*P* < 0.05 was considered statistically significant.

## 3. Results

### 3.1. Comparison of Pathogenic Microorganism Detection

#### 3.1.1. The Status of Pathogenic Microorganisms

Two methods were used to isolate pathogenic microorganisms from patients with pneumonia. The top four G^−^ detected by the two methods were *Acinetobacter baumannii*, *Klebsiella pneumoniae*, *Pseudomonas aeruginosa*, and *Escherichia coli*.

The top three G^+^ detected by the two methods were *Staphylococcus aureus*, *Streptococcus pneumoniae*, and *Streptococcus hemolyticus*. However, the number of bacteria detected by the two methods was inconsistent, as shown in Table 2. mNGS detected 3 viruses that were not detected by the traditional methods (not listed in Table 2).

#### 3.1.2. The Number of Pathogenic Microorganisms Detected

Among 180 patients with severe BP, mNGS sequencing results showed positive samples of alveolar perfusion fluid in 166 patients, while the traditional method showed positive samples in 105 patients. The positive rates of the two methods were 92.22% and 58.33%, respectively, and the difference between the two methods was statistically significant (*χ*^2^ = 55.54, *P*  <  0.001). Comparing the distribution of cases of pathogenic microorganisms detected by the two methods (0, 1, 2, and 3), it was found that the difference in the detected pathogenic microorganisms between the two groups was statistically significant (*P* < 0.001), in which the difference between 0 and 2 was the largest (NGS vs traditional method: 0:7.78% vs 41.67%, *χ*^2^ = 55.54, *P* < 0.001; 2: 50.56 vs 18.33%, *χ*^2^ = 41.38, *P* < 0.001, Table 3).

#### 3.1.3. Positive and Negative Test Results

Among the 180 patient specimens, 105 (58.33%) were found to be double positive, 14 (7.78%) were negative, and 61 (33.89%) were positive for NGS alone, and none (0.00%) were positive for the traditional method. The results of paired chi-square test showed that the difference between the two methods was statistically significant (*P* < 0.05, Table 4).

#### 3.1.4. mNGS Results of Alveolar Lavage Fluid

One patient with Gram-negative bacteria and one patient with Gram-positive bacteria were selected to show the mNGS results of common pathogenic bacteria, as shown in Figure 1. The mNGS reading rate of the patient with *Acinetobacter baumannii* infection was 5.99%. The mNGS reading rate of the patient with *Staphylococcus aureus* infection was 0.62%, which covered a high proportion of the genome.

#### 3.1.5. Distribution of Pathogens Detected by mNGS

In this study, one qualified sputum sample was extracted from each of 180 patients for bacterial culture. A total of 347 strains of pathogenic bacteria were detected and 256 strains of G^−^ were detected, accounting for 73.78% (256/347) of the total pathogenic bacteria. The top four bacteria were *Acinetobacter baumannii*, accounting for 42.19% (108/256) of G^−^; *Klebsiella pneumoniae*, accounting for 20.71% (53/256) of G^−^; *Pseudomonas aeruginosa*, accounting for 13.67% (35/256) of G^−^; and *Escherichia coli*, accounting for 11.72% (30/256) of G^−^. A total of 89 strains of G^+^ were detected, accounting for 25.65% (89/347) of the total pathogens. The top three bacteria were *Staphylococcus aureus*, accounting for 41.57% (37/89) of G^+^; *Streptococcus pneumoniae*, accounting for 35.96% (32/89) of G^+^; *Staphylococcus haemolyticus*, accounting for 10.11% (9/89) of G^+^. There were 2 strains of fungi, including 1 strain of *Candida albicans* and 1 strain of *Candida albicans*, as shown in Table 1.

#### 3.1.6. Chest CT Results of Common Bacterial Infection in Patients with Severe BP

Based on the two bacterial flora detection methods, clinicians also comprehensively determine the pathogenic pathogens related to pulmonary infection in patients based on clinical manifestations, disease evolution, patient imaging, and previous diagnosis and treatment experience. Chest CT results are shown in Figure 2.

#### 3.1.7. Analysis of Drug Resistance of Major G^−^ Bacteria

*Acinetobacter baumannii* had the highest resistance to ciprofloxacin, with a resistance rate of 80.95%. Its resistance to ceftazidime, levofloxacin, gentamicin, piperacillin/tazobactam, amikacin, and imipenem were relatively high, with resistance rates of 80.56%, 77.78%, 76.85%, 75.00%, 71.30%, and 67.59%, respectively. It had the lowest resistance to tigecycline, with a resistance rate of 4.63% only. *Klebsiella pneumoniae* had the highest drug resistance rate to piperacillin/tazobactam, with a resistance rate of 58.49%. Its resistance to ceftazidime, cefoperazone/sulbactam and imipenem were the next, with the resistance rates of 54.72%, 45.28% and 22.64%, respectively. It had the lowest resistance to amikacin, being only 3.77%.

*Pseudomonas aeruginosa* had the highest resistance to levofloxacin, with a resistance rate of 25.71%. Its resistance rates to imipenem, ceftazidime, ciprofloxacin, piperacillin/tazobactam, cefoperazone/sulbactam, and amikacin were 22.85%, 17.14%, 17.14%, 14.29%, 11.43%, and 11.43%, respectively. It had the lowest resistance to gentamicin, being 5.71%. *Escherichia coli* had the highest resistance to imipenem, with a resistance rate of 90.00%. Ceftazidime and gentamicin followed, with drug resistance rates of 85.00% and 75.00%, respectively. Its resistance to tigecycline was the lowest, with a resistance rate of 5.00%. The results are shown in Table 5.

#### 3.1.8. Analysis of Drug Resistance of Major G^+^ Bacteria

The resistance rates of *Staphylococcus aureus* to penicillin, azithromycin, amoxicillin, levofloxacin, and erythromycin were 100.00%, 94.59%, 91.89%, 70.27%, and 56.76%, respectively, among which penicillin resistance was the highest, and its resistance rates to linezolid and vancomycin were both 0.00%. *Streptococcus pneumoniae* had the highest resistance to penicillin and azithromycin, with the resistance rates being 100.00% and 100.00%. *Streptococcus pneumoniae* had low resistance to tetracycline, with a resistance of 16.63%, and its drug resistance rates to linezolid and vancomycin were 0.00% and 0.00%. The drug resistance rates of *Streptococcus hemolyticus* to penicillin, azithromycin, amoxicillin, levofloxacin, and erythromycin were 100.00%, 100.00%, 66.67%, 55.56%, and 44.44%, respectively. Its resistance rate to tetracycline was 11.11%. Its resistance rates to linezolid and vancomycin were both 0.00%. The results are shown in Table 6.

## 4. Discussion

BP is caused by pulmonary infectious bacteria and is closely related to the age, concomitant diseases, and immune status of the host. For patients with severe infection, the fatality rate of patients is high due to the severity of the disease. Moreover, the nonstandard use of antibiotics, bacterial resistance, and the change of strains has brought great challenges to clinical treatment [11]. People susceptible to BP are the elderly and children. In general, pneumonia occurs whenever the pathogen can penetrate the protective barrier of the human body to infect the lung parenchyma and overcome the host's defense mechanisms, regardless of age. However, the elderly are more susceptible to infection and are more likely to develop into severe infection due to the destruction of their defense system caused by basic diseases [12, 13]. Therefore, early identification of pathogenic bacteria can effectively improve the prognosis, improve the quality of life of patients, and has very important clinical significance for guiding clinical medication. The detection rate of microorganism identification and detection methods commonly used in clinical practice (microscopic examination and culture) is often affected by antibiotic treatment, and needs long culture time.

However, microbiological detection requires high accuracy and efficiency. Sequencing technology is a hot topic in microbial detection, especially mNGS. Unlike metagenomics, the positive predictive value of bacterial mNGS for antimicrobial susceptibility is high because all sites are basically covered, and this method can overcome the limitations of current diagnostic techniques and allow direct determination from clinical specimens. Bacterial mNGS is also faster and cheaper than other detection methods [14, 15].

According to the results of this study, mNGS is significantly superior than the traditional detection techniques in the species number of microbial pathogens detected and sensitivity (*P*  <  0.05), indicating that mNGS detection is more accurate. Adjusting the treatment plan according to mNGS test results can significantly benefit the patients, shorten the hospitalization time, and save the treatment cost. In 2017, a research team carried out a study on the application of mNGS in the diagnosis and treatment of infectious diseases and found that mNGS has higher sensitivity than traditional culture and has more obvious advantages in the diagnosis of tuberculosis, fungi, viruses, and anaerobic bacteria [16, 17].

Further analysis of antimicrobial resistance showed that a total of 347 strains of pathogenic bacteria were detected by mNGS in 180 patients in this study, including 256 strains of G^−^, 89 strains of G^+^, and 2 strains of fungi. This indicated that the distribution of severe BP pathogenic bacteria was mainly characterized by G^−^, followed by G^+^, and fungi were rare. In addition, G^−^ bacteria resistance test results in this study showed that *Acinetobacter baumannii* is an opportunistic pathogen with strong drug resistance. The drug resistance rate of *Acinetobacter baumannii* to 7 drugs was more than 60%, and the drug resistance rate of *Acinetobacter baumannii* to tigecycline was low, suggesting that *Acinetobacter baumannii* was almost resistant to all antibiotics commonly used in clinic, but the drug resistance to tigecycline was low. Tigecycline is a novel glycyrrhizin antibiotic, which has been gradually used in clinical treatment of *Acinetobacter baumannii* infection, and several studies have shown that good clinical efficacy has been achieved [18, 19]. However, some studies have shown that although tigecycline has a high bacterial clearance ability, long-term use alone may cause the emergence of drug-resistant strains and increase the culture rate [19]. The resistance rate of *Klebsiella pneumoniae* and *Escherichia coli* to ciprofloxacin was low. The reason is that the drug resistance mechanism of *Klebsiella pneumoniae*, *Escherichia coli*, and other pathogens is closely related to the ultra-broad spectrum *β*-lactamase and class C cephalosporin enzyme, and a variety of *β*-lactam antibacterial drugs can be hydrolyzed due to the drug resistance mechanism of pathogens, leading to the increasing drug resistance rate [20]. In this study, *Pseudomonas aeruginosa* had the highest resistance to imipenem and levofloxacin, its resistance to other antibacterial drugs was low, and its resistance to amikacin was the lowest. Therefore, it is not recommended to use quinolones, second-generation cephalosporins, and third-generation antibiotics alone in clinical treatment of *Pseudomonas aeruginosa* infection, and the drug combination therapy is recommended. In addition, imipenem is a common carbapenem antibiotic, which is a high-level antibiotic and can significantly inhibit the bacterial cell wall synthesis [11].

The drug resistance test results of Gram-positive bacteria in this study showed that the drug resistance rates of *Staphylococcus aureus*, *Streptococcus pneumoniae*, and *Streptococcus hemolyticus* to penicillin were all 100.00%, their resistance rates to erythromycin and tetracycline antibiotics were low, and their drug resistance rates to linezolid, vancomycin, and other antibiotics were all 0.00%. It is suggested to avoid the use of macrolides in the treatment of patients with Gram-positive bacterial infection in order to improve the clinical treatment effect.

The study also has shortcomings. The sample size was small, and the sample type was limited to alveolar lavage fluid. In the next step, the research team will expand the sample size and study refine the study groups, so as to study the mNGS technology further and improve the application value of mNGS in the diagnosis and treatment of clinical pulmonary infection.

## Figures and Tables

**Figure 1:** mNGS results of alveolar lavage fluid of two patients. (a) mNGS results of a patient with *Acinetobacter baumannii* infection and (b) mNGS results of a patient with *Staphylococcus aureus* infection.

**Figure 2:** Chest CT examination of common bacterial infection with Gram negative (positive) bacteria. (a) *Staphylococcus aureus* infection. (b) *Klebsiella pneumoniae* infection. (c) *Pseudomonas aeruginosa* infection. (d) *Escherichia coli* infection.

**Table 1:** Basic information.

Items		*N* (%)/Mean ± SD
Gender	Male	100 (55.56)
	Female	80 (44.44)

Average age (y)		55.21 ± 3.55
BMI (kg/m^2^)		22.02 ± 2.05
Average course of disease (d)		14.45 ± 2.15

**Table 2:** Distribution of pathogens identified by the two methods in BP patients in emergency intensive care unit (ICU).

Pathogens	mNGS [*N* (%)]	Traditional methods (*N* (%))
G^−^	**256 (73.78)**	**109 (74.66)**
*Acinetobacter baumannii*	108 (42.19)	60 (55.05)
*Klebsiella pneumoniae*	53 (20.71)	27 (24.77)
*Pseudomonas aeruginosa*	35 (13.67)	12 (11.01)
*Escherichia coli*	30 (11.72)	10 (9.17)
*Haemophilus influenzae*	15 (5.86)	1 (0.92)
*Stenotrophomonas maltophilia*	8 (3.12)	1 (0.92)
Others	7 (2.73)	1 (0.92)
G^+^	**89 (25.65)**	**37 (25.34)**
*Staphylococcus aureus*	37 (41.57)	20 (54.05)
*Streptococcus pneumoniae*	32 (35.96)	13 (35.14)
*Streptococcus hemolyticus*	9 (10.11)	2 (5.41)
*Enterococcus*	6 (6.74)	1 (2.70)
Others	5 (5.62)	1 (2.70)
Fungus	**2 (0.58)**	**0 (0.00)**
*Candida albicans*	1 (50.00)	0 (0.00)
Total	**347 (100.00)**	**146 (100.00)**

**Table 3:** Comparison of the species number of pathogenic microorganisms detected by the two methods (*N*(%)).

The number of pathogen species	mNGS (*N* = 180)	Traditional methods (*N* = 180)	*χ* ^2^	*P*
0	14 (7.78)	75 (41.67)	55.54	<0.001
1	30 (16.67)	68 (37.78)	20.25	<0.001
2	91 (50.56)	33 (18.33)	41.38	<0.001
3	45 (25.00)	4 (2.22)	39.71	<0.001
Total number of positive	166 (92.22)	105 (58.33)	55.54	<0.001

**Table 4:** Positive and negative detection results (*N*).

mNGS	Traditional methods		Total
	Positive	Negative	
Positive	105	61	166
Negative	0	14	14
Total	105	75	180

Note: *P* < 0.05 by McNemar test.

**Table 5:** Resistance analysis of major G^−^ bacteria.

<!—Col Count:5Antibacterial agents	*Acinetobacter baumannii*, *Klebsiella pseudomonas*, *Escherichia coli*, *and Pneumoniae aeruginosa*			
	(*N* = 108)	(*N* = 53)	(*N* = 35)	(*N* = 20)
	The number of drug-resistant bacteria (*N* (%))	The number of drug-resistant bacteria (*N* (%))	The number of drug-resistant bacteria (*N* (%))	The number of drug-resistant bacteria (*N* (%))
Cefoperazone/sulbactam	34 (31.48)	24 (45.28)	4 (11.43)	11 (55.00)
Piperacillin/tazobactam	81 (75.00)	31 (58.49)	5 (14.29)	12 (60.00)
Ceftazidime	87 (80.56)	29 (54.72)	6 (17.14)	17 (85.00)
Imipenem	73 (67.59)	12 (22.64)	9 (25.71)	18 (90.00)
Levofloxacin	84 (77.78)	8 (15.09)	8 (22.85)	10 (50.00)
Amikacin	77 (71.30)	2 (3.77)	2 (5.71)	6 (30.00)
Ciprofloxacin	85 (80.95)	7 (13.21)	6 (17.14)	3 (15.00)
Gentamicin	83 (76.85)	3 (5.66)	4 (11.43)	15 (75.00)
Polymyxin B	12 (11.11)	—	—	—
Minocycline	10 (9.26)	—	—	2 (10.00)
Tegacyclin	5 (4.63)	—	—	1 (5.00)

**Table 6:** Resistance analysis of major G^+^ bacteria.

Antibacterial agents	*Staphylococcus aureus* (*N* = 37)	*Streptococcus pneumoniae* (*N* = 32)	*Streptococcus hemolyticus* (*N* = 9)
	The number of drug-resistant case (*N* (%))	The number of drug-resistant case (*N* (%))	The number of drug-resistant case (*N* (%))
Penicillin	37 (100.00)	32 (100.00)	9 (100.00)
Linezolid	0 (0.00)	0 (0.00)	0 (0.00)
Azithromycin	35 (94.59)	32 (100.00)	9 (100.00)
Erythromycin	21 (56.76)	19 (59.38)	4 (44.44)
Vancomycin	0 (0.00)	0 (0.00)	0 (0.00)
Amoxicillin	34 (91.89)	25 (78.12)	6 (66.67)
Levofloxacin	26 (70.27)	21 (65.63)	5 (55.56)
Tetracycline	7 (18.92)	5 (15.63)	1 (11.11)

## Data Availability

The data used in this study are available from the corresponding author upon request (Fanguofeng98@163.com).
